# Biological Breakdown of Sports in Athletics Based on Multimedia Image Acquisition Techniques

This article has been retracted.

**DOI:** 10.1155/2022/3497942

**Published:** 2022-03-29

**Authors:** Peng Sun, Biyu Zhang, Qiaoling Chen, Jianbang Guo

**Affiliations:** ^1^Beijing Sport University China Athletics College, Beijing 100084, China; ^2^Anqing Normal University Physical Education College, Anqing, Anhui 246133, China; ^3^Capital University of Physical Education and Sports, Beijing 100091, China

## Abstract

This paper provides an in-depth analysis and study of the decomposition of sports biology of athletics events through multimedia image acquisition techniques. The proposed design uses SOPC hardware-software collaboration technology, which makes full use of the parallelism of hardware as well as the flexibility of software to essentially improve the speed of image processing and greatly improve the efficiency of image processing. The high speed and parallelism of hardware are used to realize the image acquisition part with high timing requirements and the preprocessing algorithm with a large number of operations and strong repetition, in addition to the difficulties of many initialization configuration parameters of each peripheral. Additionally, the need for frequent adjustment of peripheral working parameters is solved by making full use of the scalability and flexibility of software, and the control signals output by software can coordinate the work of each hardware module to ensure that each module of the system cooperates. It is also possible to coordinate the work of each hardware module through the control signal output from the software to ensure that each module of the system cooperates and operates in an orderly and efficient manner and provides the possibility of realizing a higher level of the image processing algorithm. The system includes four main factors: swinging action, supporting action, vacating action, and speed rhythm. Based on this system, 14 key kinematic indicators were selected to reflect the technical status of the youth walkers. The landing angle decreased with the increase of speed, and the landing technique was insufficient; it had better control of the large and small arm angle, and their stride width was open, while the other four athletes showed increased tension in the hip joint and upper limb with the increase of walking speed, as well as the wrong action of forward and internal rotation of the large and small arms.

## 1. Introduction

The globalization of knowledge and the rising tide of scientific and technological innovation have made innovation capabilities the main driver of competitive advantage for technological agents. The creation and flow of knowledge are a key factor for national economic growth at the macro level while determining the competitiveness of scientific research at the micro level [1]. Against the background of accelerated technological change and knowledge flow, global knowledge subjects gradually present a state of open development of interconnection, interdependence, and competition among themselves [2]. The way for organizations to accelerate the pace of innovation and enhance innovation capacity has also shifted from mainly independent research to technology alliances, external acquisition, and other channels. The aim is to achieve sustainable development of competitiveness by tapping effective external innovation resources through imitation, cooperation, and learning. An important way for scientific research-related institutions and personnel to acquire external knowledge, improve innovation capabilities, and upgrade their position is generated in the process of knowledge flow, which is an important source of maintaining long-term competitive advantage in scientific research. As the quality of life of people is getting better, the impact of image surveillance and image recognition on people's lives is increasing [3]. A prerequisite for image processing is to first acquire high-quality images, and image acquisition devices are generally used as the front end of image processing. The raw image data provided will be sent to the image processing module, or the acquired image data can be stored first, buffered, and then removed for image processing at the end. Image acquisition and image processing together form a complete system that can be widely used in important areas such as medical detection, agricultural detection, and security monitoring. It can be said that the merit of image acquisition is an important criterion for judging the quality of image processing.

The rapid development of optical remote sensing technology has not only laid the foundation for humankind to obtain stronger and stronger Earth observation capability but also provided favorable support and guarantee for various application fields closely related to human life. However, the rapid development of remote sensing technology has also brought about an explosive growth of remote sensing data volume. Therefore, how to decode the massive remote sensing data intelligently and rapidly and how to extract useful key information from these massive multisource heterogeneous remote sensing data have become an inevitable requirement in the era of remote sensing big data [4]. Given that different types of optical remote sensing data acquired by different sensors not only have their data characteristics but also have different feature distribution characteristics, different interpretation strategies and methods should be applied to different types of optical remote sensing data. The concept of action measurement feedback refers to the use of relevant technical equipment in the process of each technical action operation, the technical action is filmed and tested for relevant indicators, and the appropriate feedback is given to the students at the right time, and the students observe and control the relevant indicators, to promote the improvement of skills. The proposed feedback for measurements of actions is based on the derivation of positive feedback, negative feedback, and self-feedback in physics. In this study, the difference from other assessment feedbacks is that the content of the movement assessment feedback is the key numerical indicator of specific movements and the students adjust the relevant technical movements by observing the changes of the values. Additionally, the selection of key indicators depends on the requirements of relevant technical movements. In addition, the feedback method is continuous process feedback in the process stages.

Students' feedback in the movement assessment feedback process comes from feedback sheets, peers, and teachers, and students adjust and change in technical movements based on the changes in values in the feedback sheets, a process in which students continue to explore the effectiveness of the movements. The movement assessment feedback in this feedback emphasizes the process of giving students precise numerical categories of change in stages of instruction, presenting the process of change in numerical form. An attempt is made to encourage students to take the initiative to think, to play the role of the student and the role of the teacher, and ultimately to achieve the reinforcing effect of combining internal and external aspects. Logical functional simulation of the designed logic circuit, in which there is no delay information to verify that the designed logic circuit meets the requirements of the design, is an important part of the design and affects the development cycle of the design, applying ModelSim simulation tool to complete the functional simulation. The logic circuit after the functional simulation is synthesized and optimized, and the complex logic circuit is synthesized into a netlist consisting of gate circuits and flip-flop units, which is done by the development tool that comes with the FPGA to make the designed logic circuit more specific. The postsynthesis simulation is used to see if the synthesized circuit is consistent with the design goals. Current synthesis tools are more mature and this step can generally be omitted. Configure the synthesized and optimized logic netlist into the corresponding development chip, and use the internal connectivity resources of the chip to optimize the speed and area through a reasonable layout and wiring. The delay information after layout and wiring is marked into the design netlist to determine whether there are timing violations in the logic design and to reduce the possibility of generating competition and risk by analyzing the timing of the design logic modules and performing timing constraints. Board-level simulation is commonly used in high-speed logic circuit design, mainly to check the signal integrity of the circuit, electromagnetic interference, and so forth. In most cases, third-party simulation verification tools are utilized.

The main contributions of this study are as follows:

- Movement assessment feedback mechanism for students which are useful in adjusting a relevant movement preferably technical.
- A methodology which is very helpful for students to take initiative in thinking, playing numerous roles such as student and teacher, and reinforcing internal and external aspects to achieve the required aspects.

The remainder of the paper is organized as given below.

In the subsequent section, a brief review of the most relevant literature is presented along with identification of the various issues associated with these approaches. In Section 3, multimedia image acquisition technique is described in detail which is followed by experimental results and observations, preferably both in textual and graphical formats. Finally, concluding remarks are given at the end.

## 2. Current Status of Research

In the process of face image acquisition, the synchronization of image acquisition has a large impact on the modeling accuracy, so it is necessary to study the synchronization control method of image acquisition [5]. The synchronization control method of multiple images is divided into software synchronization and hardware synchronization; software synchronization is to use software to send acquisition commands and generate synchronization trigger signal by external synchronization signal generator to control multiple image acquisition devices to synchronize acquisition; this method requires the high performance of synchronization trigger signal. Hardware synchronization is to connect the trigger master controller with the image acquisition device through the hardware synchronization chip and use the synchronization trigger signal generated by the synchronization chip to realize the acquisition of multiple images, and the commonly used hardware synchronization methods are multiple image data acquisition cards, multiple peripheral component interconnect (PCI) bus data acquisition cards, and external trigger signal source data acquisition cards [6]. Among multiple image data acquisition cards, for high-resolution images, image data volume is large; when multiple image data acquisition cards work together, there are large data transmission bandwidth requirements for the transmission line. Multi-PCI bus data acquisition cards need PCI data acquisition card drivers to complete the synchronization control between multiple PCI cards; the method requires strong programming skills [7]. The most important thing to remember about the various motor skill learning models is that they are not superior or inferior in value [8]. No motor skill learning model is better than the others, and no group of styles can stand alone; they complement each other and influence each other, but each has a greater or lesser role to play, and the best should be taken and the worst removed. In the actual teaching of motor skill learning styles, teachers should assess the learning styles of their students so that they can tailor their teaching to suit their needs.

Tan Jian Gong believes that the transition process from the preswing phase to the spin phase plays an important role in the transition of the chain ball to the spin phase [9]. If the athletes' technical movements are reasonable in this process, the transition from preswing to spin phase will become tight and will bring a good rotation rhythm to the spin phase to guarantee the ideal throwing performance. However, if the chain ball does not move correctly from the preswing phase to the spin phase, then even if the spin technique is used properly, the best throwing results will not be achieved [10]. Therefore, the ideal technique for the transition from the preswing phase to the spin phase is to gradually shift the weight to the left leg and lock the left side to control the ball as much as possible. If the athlete can do this, the result will be a strong and smooth progression into the spin phase. Although the above learning models produce approximately the same results, the differences embedded in them are quite profound and the resulting instructional outcomes vary widely [11]. In the past, the research was fruitful, but the authors also found places that can be enriched: among them, some scholars believe that we should encourage the establishment of a diverse evaluation system to improve the original system. We should also avoid a single evaluation system and fixed evaluation methods, system changes can help students develop the habit of lifetime physical education. Mixed learning model puts more emphasis on the learner's mastery of the learning content, so that it causes relatively single form of interaction between teachers and students, while this interaction should be enriched and diversified during the actual teaching process; in addition to the objective needs, the experimental subjects in some studies also need a certain level of technology as a prerequisite; past studies given to students are also only animation, images, and other nonquantitative, nonobjective information; these unfavorable factors to a certain extent are held back in the actual teaching [12]. Therefore, we believe that these constraints can be improved by changing the method.

An important way for knowledge to create value lies in the flow and sharing of knowledge, and how to survive and thrive better in a complex, changing, and dynamic environment is one of the important issues facing enterprises. Knowledge becomes the most important resource for enterprises to compete. Knowledge transfer plays the most crucial role in this process. Interenterprise knowledge transfer is the process of knowledge flowing between different knowledge systems. This process is influenced by factors such as the direction, content, quantity, and path of knowledge transfer, which is a dynamic and multidimensional complex process.

## 3. Multimedia Image Acquisition Techniques to Assist in the Analysis of the Biological Breakdown of Sports in Track and Field Events

In this section, a detailed description of the proposed approach is presented, that is, multimedia image acquisition approach which is especially designed for the analysis of the biological breakdown of sports in various events related to field and track. Initially, a detailed description of the technology, which is used to capture high-quality images, is presented.

### 3.1. Design of Multimedia Image Capture Technology for Athletics

In the analysis and interpretation of optical remote sensing images, the region of interest detection technique has received a lot of attention from researchers because it enables the fast extraction of key feature information in remote sensing images by quickly locating the feature targets of interest in large-format remote sensing images [13]. In this paper, the research on the feature of interest target detection is based on the premise of detecting a feature of interest targets in images based on the visual saliency model established by visual attention mechanism without any target a priori and task-driven. This section will focus on two representative visual saliency models and analyze their suitability for application on remote sensing images from both algorithmic theoretical and experimental perspectives, thus laying the foundation for establishing the focus and goals of the subsequent research content. Developers should first go to analyze the requirements of the project and then divide the tasks and functions of each module [14]. After the division is done, the detailed design including code implementation, comprehensive optimization, and implementation (layout wiring and timing constraints and simulation) is then carried out. To confirm whether the designed effect can meet the expectation, behavioral simulation is needed during code implementation, functional simulation of the design is needed after synthesis optimization, and simulation verification of timing is needed to be completed after implementation. The final step is board-level debugging, where the EDA tool checks for errors and then creates the downloaded configuration file and burns it into the FPGA chip. From a broad perspective, the FPGA development process can be broadly divided into three phases [15]. The first phase is the architecture design phase, which is intended to prepare the project, analyze the project requirements, and delineate the functionality of each designed module. The second phase is the design implementation phase, which includes writing RTL code and performing initial functional verification, logic synthesis, layout wiring, and timing violation checks; the third phase is the FPGA implementation phase, which should include layout wiring and timing verification in addition to program download (device burn-in) and board-level debugging. In terms of the phases, the various steps in the FPGA development process are not independent of each other but are closely related and affect each other, as shown in Figure 1.

Therefore, from the experimental results, the classical saliency model applicable to natural images does not apply well to remotely sensed images. The reason for this is mainly that there is any inconsistency between the original intention of the algorithm design and the region of interest detection needs of remote sensing images. Taking the CA model as an example, in most of the spatial domain saliency models, the appearance contrast based on color features plays an important role in the saliency model, but, for optical remote sensing images with intricate feature structures, it is difficult to extract the feature targets of interest effectively from them by the contrast on color features alone [16]. Especially for panchromatic remote sensing images with no feature color at all, it is difficult to obtain high-quality detection results of regions of interest using such a saliency model. In addition, the CA model enhances the saliency detection results by introducing central prior knowledge to emphasize the region near the image center. However, in remote sensing images, the distribution of the features of interest usually has little regularity and is not concentrated in the center of the image or far from the boundary regions of the image but is scattered randomly over the entire magnitude of the remote sensing image.

(1) $$\begin{array}{c} d\left(p_{i},p_{j}\right)=\frac{d_{\text{color}}\left(p_{i},p_{j}\right)}{1-c\cdot d_{\text{color}}\left(p_{i},p_{j}\right)},\\ S_{i}=1+\exp\left\{\frac{1}{K}\sum_{k=1}^{K}d_{\text{color}}\left(p_{i},p_{j}\right)\right\}. \end{array}$$

Furthermore, considering that image blocks in the background region are similar at multiple scales; in contrast, image blocks in the saliency region may be similar at only a few scales but not at all scales. Therefore, multiple scales may be used to further reduce the saliency of background pixels and enhance the contrast between salient and nonsalient regions.

(2) $$\begin{array}{c} S_{i}^{T}=1+\exp\left\{\frac{1}{K}\sum_{k=1}^{K}d_{\text{color}}\left(p_{i}^{T},p_{j}^{T}\right)\right\}. \end{array}$$

Finally, according to the criterion, the significance detection results can be further enhanced by incorporating prior knowledge of the significant region in the derived significance estimation results. It is known that people take pictures to frame the target of interest at a location near the image center. Therefore, the region near the center of the image can be emphasized by introducing Gaussian descent weights to better predict the significant targets in the image. By incorporating a central prior in the saliency estimation model, more accurate saliency detection results can be obtained.

(3) $$\begin{array}{c} G_{i}=\exp\left\{\frac{1}{K}\sum_{k=1}^{K}d_{\text{color}}\left(p_{i}^{T},p_{j}^{T}\right)+w_{i}\right\}. \end{array}$$

Unlike the spatial domain saliency models, the transform domain-based saliency models need to first transform the image from the spatial domain to the frequency domain, then process and analyze the image in the frequency domain, and finally obtain the final saliency detection results by transforming the analysis results in the frequency domain back to the spatial domain. The most representative saliency calculation models in this type of method are the proposed spectral residual (SR) saliency model and the proposed Fourier transform (PFT) domain phase spectrum based saliency model. Here we take the PFT model as an example to introduce the transform-domain saliency model [17]. For a two-dimensional signal like an image, the resulting image amplitude spectrum clarifies the percentage of each sinusoidal component by performing the Fourier transform on it, while the phase spectrum of the image gives the position of each sinusoidal component in the image. In the reconstruction of the image in the Fourier transform domain, the positions located in the horizontal or vertical directions with weak periodicity or homogeneity correspond to the positions of the candidate targets in the image, and thus it is known that the saliency information of the image is implicit in the phase spectrum of the image. Therefore, the saliency detection result of an image can be obtained by extracting the phase spectrum information of the image. For a given image, the Fourier transform is first applied to it, thus transforming the image from the spatial domain to the frequency domain.

(4) $$\begin{array}{c} F\left(f\left(x,y\right)\right)=F\left(f\right)\left(u^{2},v^{2}\right),\\ p\left(u,v\right)=\text{angle }F\left(f\right)\left(u^{2},v^{2}\right). \end{array}$$

Next, by performing an inverse Fourier transform on the phase spectrum information of the image, the result containing the image saliency information is output in the spatial domain. From the above analysis, the PFT transform domain saliency detection model has the advantages of simple and easy algorithm and fast operation, thus giving fast saliency detection results for a given image, but the disadvantage is that it does not consider the local saliency features of the image and lacks suitable biological psychological support and explanation.

Therefore, from the experimental results, the classical saliency model applicable to natural images does not apply well to remotely sensed images. The reason for this is mainly that there is any inconsistency between the original intention of the algorithm design and the region of interest detection needs of remote sensing images. Taking the CA model as an example, in most of the spatial domain saliency models, the appearance contrast based on color features plays an important role in the saliency model, but, for optical remote sensing images with intricate feature structures, it is difficult to extract the feature targets of interest effectively from them by the contrast on color features alone. Especially for panchromatic remote sensing images with no feature color at all, it is difficult to obtain high-quality detection results of regions of interest using such a saliency model. In addition, the CA model enhances the saliency detection results by introducing central prior knowledge to emphasize the region near the image center. However, in remote sensing images, the distribution of the features of interest usually has little regularity and will not be concentrated in the center of the image or far from the boundary regions of the image but scattered randomly over the whole magnitude of the remote sensing image, as shown in Figure 2.

The objective evaluation method for the region of interest detection is to assess the merit of the region of interest detection results and the performance of the detection algorithm based on the manually annotated real region of interest. The commonly used objective evaluation metrics are accuracy rate, completion rate, F-measure value, and area under the receiver operating characteristic curve. The accuracy rate is the proportion of the number of samples that are correctly detected as the true sense region of interest out of the total number of samples contained in the detected region of interest. There may be two cases in the actual detection process; that is, it is possible to detect the samples of the true sense region of interest as the region of interest, which is called a true case, and it is also possible to detect the samples of the nontrue sense region of interest as the region of interest, which is called a false-positive case. Through the above analysis of athlete selection in each country, we can see that the pattern of athlete selection has a lot to do with the system and the importance of each country. Even though there are differences in the selected models of each country, the essence is the same; that is, they all test the athletes' morphology, function, quality, technology, and psychology through observation and scientific testing index system among many children and teenagers to select excellent athletes at different levels. From the perspective of the importance of athlete selection in the world's major competitive sports powers, the start is relatively late, but the development speed is fast, and the current theoretical system is relatively mature, and a perfect selection index system and evaluation standards for each project have been established. All these have laid the foundation for the rapid development of China's competitive sports and provided a reliable talent guarantee for China's competitive sports to continue to compete on the same field with the world powers such as Europe and America.

### 3.2. Experimental Analysis of the Biological Breakdown of Movement in Track and Field Events

The 20 km race walk is a long-distance, long-time, and physically demanding sport, and it takes time for the athletes to enter the race and overcome the poles at the beginning of the race, as shown in Figure 3. The speed at the beginning of the race is slow. In the middle of the race, athletes need to maintain their physical fitness to continue the race, and the speed fluctuation is small, to maintain physical fitness at medium speed [18]. The latter part of the race starts with varying degrees of speed to gain a place in the race. The average speed of the six athletes in the first ten laps was 4 : 09 min/km and the average speed in the second ten laps was 4 : 04 min/km. In the last stage of the race (lap 20), some athletes with better fitness, such as Wang Kaihua, Bian Tongda, and Yang Liang, were able to sprint at a higher speed. The characteristics of speed change in this race are consistent with the study of the world's best men's 20 km race walkers who have slow speed in the front and fast speed in the back. The average speed of the six athletes in laps 3 and 4 is 4 : 15 min/km, and laps 3 and 4 are the low-speed laps of each athlete, so the horizontal comparison of the six athletes and the vertical comparison of each athlete are reasonable [19]. The technical movements of laps 3 and 4 are selected as the low-speed range.

The speed of the top six athletes accelerated in lap 5 and remained relatively stable until lap 13, and the overall trend showed that the top six athletes walked at medium speed in lap 6. The average speed of the first six athletes in lap 6 was 4 : 05 min/km which was less different from the average speed of 4 : 07 min/km; after lap 6, the speed of the six athletes changed a lot and could not be compared at the same speed, so the first six athletes were chosen to analyze the technical movements in the medium speed interval in lap 6. Except for Wang Qin, whose high speed appeared earlier, the other five athletes tended to increase their speed in laps 13 and 14, and the highest speed appeared in lap 12 at 4 : 00 min/km. Yang Liang's high speed appeared later, accelerating at lap 15 and decreasing after lap 15, with a maximum speed of 3 : 54 min/km on lap 20. The speed was higher on lap 15 and the highest speed was 3 : 51 min/km on lap 20, so lap 20 was chosen as Wang Kaihua's high-speed interval.

The start-rotation technique is the transition of the chain ball from the preswing phase to the rotation phase. Its main function is to make a smooth transition from the speed obtained in the preswing phase to the rotation first turn, to ensure that the chain ball has the proper rotation initial speed when it enters the rotation phase. At the same time, the starting rotation technique contains the double support phase in the first revolution of rotation, and there are relevant studies that show that the double support phase during rotation is the main acceleration phase of the chain ball, and to make the chain ball movement able to be continuously accelerated, the time of the double support phase should be increased as much as possible. Therefore, based on obtaining a larger ball speed in the preswing phase, try to grow the force-time of the starting rotation technique and increase the action distance to ensure the continuous acceleration of the chain ball in the rotation phase. We can see that the average time taken by the four players in the start-spin technique is 0.77 s, with a standard deviation of 0.05 s; that is, the time taken by the four players in the start-spin technique is relatively small [20]. The time spent on the starting technique is longer by Wang Zheng and Liu Tingting; both of them spend 0.80 s on the starting technique, but the time spent in the starting technique by Wang Zheng accounts for 17.97% of the total time, and the time spent in the starting technique by Liu Tingting accounts for 15.37% of the total time; the difference between the time spent in the starting technique and the total time is 2.60%, which means that the time spent in the starting technique by Wang Zheng in the complete chain ball throw is relatively longer. However, the time spent by Rona in the start and turn technique accounted for 14.52% of the total time spent, which was 2.02% greater than the time spent by Zong Dan in the start and turn technique, indicating that Rona's start and turn technique accounted for a greater proportion of the total time spent in the chain toss compared with Zong Dan, as shown in Figure 4.

The human body goes through two periods of growth and development, and the adolescent period is in the second period of life, due to the rapid development of various indicators such as physical form, function, and quality; therefore, in the process of selecting athletes, the selection criteria should be formulated according to the development and project characteristics in line with the different age groups, and, secondly, the age characteristics of training methods and means should be paid attention to in this period, that is, more emphasis on aerobic training. In addition, the relationship between nutrition, training, and rest for athletes in this age group should be handled. Some systems develop earlier, such as the nervous system, while others develop later, such as the reproductive system. Therefore, we should fully consider the unbalanced development of the nervous system in the process of selecting and nurturing athletes, pay attention to the screening and selection of the nervous system in the early stage of athletes, and pay attention to the improvement of the function of the nervous system of athletes in the early stage, such as sensitivity, coordination, sense of rhythm, and other abilities that are more related to the nervous system.

The so-called believed law refers to the centripetal pattern of body form in the process of growth and development. Development is characterized by the following: lower limbs before upper limbs, limbs before trunk, bottom-up, and from the distal end of the limbs to the center trunk development pattern. This inspires us in the selection process of young people that we should develop selection criteria that meet the common characteristics of different age groups according to their growth and development characteristics.

## 4. Analysis of Results

### 4.1. Results of Multimedia Image Acquisition for Athletics

In this paper, we build the hardware environment of the multichannel image synchronous acquisition system and complete the logic design of each module of the system, which mainly includes the multichannel image synchronous acquisition module, image data cache module, image preprocessing module, HDMI display module, and Ethernet transmission module. The hardware is shown in Figure 5. The FPFA chip XC7A100T is used as the control core, CMOS OV5640 is used as the image data acquisition terminal, DDR3 SDRAM is used for image data caching, HDMI interface is connected to HDMI display to complete the image display, and Ethernet interface realizes the image data transmission. The logic design of each module of the system has been simulated in Chapter 3, and the test results show that the logic design is correct. After power-on reset, the FPGA controls the CMOS OV5640 to capture multiple images, the DDR3 SDRAM to cache the image data, and the HDMI display of the images. At the same time, the images are transferred to the PC via Ethernet to complete the image saving. Then, we carried out practical tests on the test board for each submodule separately, and the results met the design requirements. The group conducted the overall functional test of this acquisition system, and the HDMI display results are shown in Figure 5. Figure 5 shows the single-channel face image captured with a resolution of 1280 × 720. Figure 5 shows the dual-channel face image captured with CMOS1 on the left and CMOS2 on the right, with a resolution of 640 × 720. As can be seen above, the face image captured by the camera can be displayed correctly on HDMI, indicating that the designed multichannel image synchronization acquisition system meets the design requirements.

The image blur detection algorithm proposed in this paper can effectively detect the blurred images and the detection accuracy reaches 90.13%. The reason for higher detection accuracy than that the proposed algorithm is that the detection accuracy obtained by the edge-based blur detection algorithm is the lowest due to the small number of edges contained in the face. When an all-black image or a blurred image is acquired, the image is not available, resulting in low accuracy of the 3D face model generated later. All-black image detection and blur detection are added to the image preprocessing module for rejecting the captured all-black images or blurred images, thus improving the efficiency of the system.

The two groups were evaluated before and after the experiment, using the Sony FDR-AX100E HD video camera at 100 frames per second to shoot the testers in action, and the video taken by the camera was processed by Kinovea software to give feedback to the athletes when the shooting was completed, and the final data is presented in Figure 6; both the experimental group and the control group showed an increasing trend, and the experimental group also had only a small advantage in the last test. Reviewing the overall data changes, it is easy to find that the control group is always in the overall development of the “wave” in the substantial difficulties, as well as high uncertainty and unmanageability; compared to the experimental group in the overall trend of a steady rise, the process also has a decline but only a small decline in the steady growth of the “debugging state.” In summary, although the final test results of the experimental group and the control group were nearly similar, the process data of the experiment showed that the experimental group was more controllable than the control group, and the experimental group would “instinctively” review the previous movement technique and the process details of the throw after comparing the previous experimental data, and this process is precisely a review of the movement. This process is precisely a review of the movement, thus achieving the desired effect of a steady stepwise increase in the data. The overall comparison increases the teacher's control over the student's performance and learning status at this stage, thus maximizing the educational impact.

In addition to the verbal community, the movement community is another aspect that cannot be ignored. The number of experimental groups in the process of observing and imitating others' throws was significantly higher than the number of control groups, and it is believed that the practitioners recognized the importance of technical movements for performance improvement while focusing on performance; the authors found that among the practitioners waiting for the test in the same test conditions the experimental groups would form small discussion groups of 2–3 people, all sharing the same procedural nature. When the others were ready to throw, they were discussed and observed together. When the others were about to throw, the discussion decreased. During the throw, the observers looked up and followed the ball until it landed. After landing, they discussed again or some of them imitated the action.

### 4.2. Experimental Results on the Biological Breakdown of Movement in Track and Field Events

According to the clustering structure of the tree diagram, at 15–20, the keyword clustering structure can be divided into 4 class clusters, which is close to the results of the multidimensional scale analysis method. For a more detailed analysis, it is possible to broadly classify the research topics on the sources of knowledge absorption in athletics into 11 class clusters based on distances 10–15. Class 1 is related to research on the issue of blood lactate accumulation. Category 2 is concerned with the analysis of aerobic capacity in elite athletes over long distances. Category 3 is research related to endurance issues in middle- and long-distance athletes. Category 4 is related to studies on maximal oxygen uptake in power cycling. Category 5 is about studies related to the physiological mechanisms of anaerobic exercise in athletes. Category 6 is about the analysis of skeletal muscle glycogen problems. Category 7 is about studies related to blood loss during exercise. Category 8 is about studies on serum, creatine kinase, testosterone, and other issues. Category 9 is about studies on the acute response of the athlete's sprinting heart. Category 10 is about cardiac coronary artery-related studies. Category 11 is about studies related to bone density and body mass, as shown in Figure 7.

Based on the consultation with experts, the psychological questionnaire was used to test the psychological characteristics of middle and long-distance runners, and the testing process tried its best to exclude interference and difficult factors to ensure the accuracy of the data. Through statistical analysis of the actual measured values of the psychological characteristics of women in group A, there were no statistically significant indicators between the athletes in the excellent group and the general group. All the psychological test indicators of this group were subjected to factor analysis, and, before factor analysis, Kaiser-Meyer-Olkin (KMO) and Bartlett tests were first conducted on the physical function indicators of the athletes in this group, and the test results showed that the KMO statistic was greater than 0.5 and Bartlett spherical test, and the original hypothesis of unit correlation matrix was rejected, as shown in Figure 8.

The results show that there are 4 factors with eigenvalues greater than 1, namely, 1500 m, standing triple jump, sitting forward bend, and 1 min alternate feet jump rope, and the cumulative contribution of the 4 factors is 78.978%, which includes the statistical screening of the actual test values between the excellent group and the general group. 1500 m mainly reflects the endurance quality of athletes, which can effectively reflect the general endurance level of middle- and long-distance runners. The 1500 m mainly reflects the endurance quality of athletes, which can effectively reflect the general endurance level of middle- and long-distance runners; the standing triple jump index can reflect the explosive power and bouncing power of athletes' lower limbs and even the coordination of athletes; the seated forward bend index can reflect the flexibility quality of middle- and long-distance runners; the 1 min double foot alternating rope skipping can reflect the coordination of athletes, which is found to be poor in the actual test process. 4 factors are consistent with the characteristics of the physical quality items of athletes in this group and are suitable. The four factors are consistent with the characteristics of the physical quality items of the athletes in this group and are suitable as the selection index of the physical quality of the athletes in this group.

For maximum oxygen uptake/body weight index, maximum oxygen uptake reflects the amount of oxygen that can be taken per unit time when the human body has a large number of muscle groups involved in exercise; when the cardiorespiratory function and the ability of muscles to use oxygen reach the limit level of the human body, generally use its relative value for interindividual comparison; for red blood cell index, red blood cells have the role of transporting oxygen, carrying oxygen, exercise dioxide, and buffering blood acidity; the number of red blood cells is related. The erythrocyte count is related to the sport, and the total number of erythrocytes is generally higher in middle- and long-distance runners, but the increase in the number of erythrocytes per unit volume is not obvious; hemoglobin index can be used to assess the functional status of athletes, and this index is mainly used in aerobic work-based events, and it is an important reference value for the selection of athletes for endurance and speed endurance events. The three common factors of the factor analysis results are consistent with the characteristics of middle- and long-distance running events and are suitable as indicators for the selection of athletes' physical performance in this group.

## 5. Conclusion

An image denoising algorithm was completed for image quality degradation caused by the introduction of noise in the image acquisition process. The image contrast enhancement algorithm research was completed for the case of insufficient image contrast caused by insufficient external light or overexposure. Considering the existence of feature extraction in the later 3D face modeling, the image edge detection algorithm research was completed. Using the FPGA parallel processing capability, the FPGA implementation of fast median filtering, histogram equalization, and Sobel edge detection algorithm of the image was completed, reducing the processing time on the PC side in the later stage. Although the experimental group was ahead of the control group in 5 of the 8 distances' data, the overall effect was not significant. However, the experimental group was higher than the control group in terms of the overall level of skill learning, technical normality, and skill rating. Therefore, the experiment proves that the method cannot achieve significant growth in the distance in the short term, but it is effective in skill assessment and can improve the normality, stability, and accuracy of motor skills. It is believed that it is the change of feedback pathway and feedback method that improves teaching quality under the same number of teaching times. Movement assessment feedback can effectively improve the quality of the teaching process, improve the standardization of movements, and significantly improve students' quality of will and sense of experience, which indicates that process feedback is beneficial for short-term course teaching, and proving its long-term effects needs further experiments.

## Figures and Tables

**Figure 1:** Development flow chart.

**Figure 2:** Functional block diagram.

**Figure 3:** Top six-segment speeds.

**Figure 4:** Experimental steps.

**Figure 5:** Detection accuracy.

**Figure 6:** Velocity phase change diagram.

**Figure 7:** Absorbing source subject keywords.

**Figure 8:** Indicator factor analysis variance contribution.

## Data Availability

The datasets used and/or analyzed during the current study are available from the corresponding author upon reasonable request.
